The article "Effect of Interventional Therapy on Iliac Venous Compression Syndrome Evaluated and Diagnosed by Artificial Intelligence Algorithm-Based Ultrasound Images" was published in 2021. Journal: J Healthc Eng.

# Effect of Interventional Therapy on Iliac Venous Compression Syndrome Evaluated and Diagnosed by Artificial Intelligence Algorithm-Based Ultrasound Images

**DOI:** 10.1155/2021/5755671

**Published:** 2021-07-22

**Authors:** Ye Bai, Fei Bo, Wencan Ma, Hongwei Xu, Dawei Liu

**Affiliations:** ^1^Department of Interventional Operating, Chengde City Central Hospital, Chengde 067000, Hebei, China; ^2^Department of Ultrasound Diagnosis, Chengde City Central Hospital, Chengde 067000, Hebei, China; ^3^Department of Radiology, Chengde City Central Hospital, Chengde 067000, Hebei, China; ^4^Department of Interventional Vascular Surgery, Chengde City Central Hospital, Chengde 067000, Hebei, China

## Abstract

In order to explore the efficacy of using artificial intelligence (AI) algorithm-based ultrasound images to diagnose iliac vein compression syndrome (IVCS) and assist clinicians in the diagnosis of diseases, the characteristics of vein imaging in patients with IVCS were summarized. After ultrasound image acquisition, the image data were preprocessed to construct a deep learning model to realize the position detection of venous compression and the recognition of benign and malignant lesions. In addition, a dataset was built for model evaluation. The data came from patients with thrombotic chronic venous disease (CVD) and deep vein thrombosis (DVT) in hospital. The image feature group of IVCS extracted by cavity convolution was the artificial intelligence algorithm imaging group, and the ultrasound images were directly taken as the control group without processing. Digital subtraction angiography (DSA) was performed to check the patient's veins one week in advance. Then, the patients were rolled into the AI algorithm imaging group and control group, and the correlation between May–Thurner syndrome (MTS) and AI algorithm imaging was analyzed based on DSA and ultrasound results. Satisfaction of intestinal venous stenosis (or occlusion) or formation of collateral circulation was used as a diagnostic index for MTS. Ultrasound showed that the AI algorithm imaging group had a higher percentage of good treatment effects than that of the control group. The call-up rate of the DMRF-convolutional neural network (CNN), precision, and accuracy were all superior to those of the control group. In addition, the degree of venous swelling of patients in the artificial intelligence algorithm imaging group was weak, the degree of pain relief was high after treatment, and the difference between the artificial intelligence algorithm imaging group and control group was statistically considerable (*p* < 0.005). Through grouped experiments, it was found that the construction of the AI imaging model was effective for the detection and recognition of lower extremity vein lesions in ultrasound images. To sum up, the ultrasound image evaluation and analysis using AI algorithm during MTS treatment was accurate and efficient, which laid a good foundation for future research, diagnosis, and treatment.

## 1. Introduction

Iliac vein compression syndrome (IVCS) is called Cockett syndrome and May–Thurner syndrome. It is a disease of physiological changes such as changes in the venous pressure of the lower extremities and venous return disorders caused by continuous compression of the iliac veins, which is also a common disease in clinical vascular disease [1]. In the early 1957, May and Thurner first proposed the anatomical basis of IVCS through autopsy research. Since the position of the iliac vein is different from the usual anatomy, the left common iliac vein receives the pressure of the bone and the stimulation of the blood vessels from the right common iliac artery and the lumbar spine. Compression of the left common iliac vein is the most common clinical case [2–4]. In addition, other general factors such as abdominal aorta, bladder disease, local kidney, pelvic tumor, and other high branches would also put pressure on the iliac vein [5–7]. The most important methods for detecting IVCS include ultrasound, computed tomography (CT), magnetic resonance imaging (MRI), and positron emission tomography (PET) [8–11]. To save time and money, ultrasound has become the first choice for IVCS. However, the iliac vein compression point is combined with the surrounding mechanism in the ultrasound image of IVCS, which is difficult to distinguish with the naked eye. Due to the various experiences of doctors, needle biopsy, ablation, and other surgical treatment methods are used for various diagnostic results. Sometimes when surgery is not needed, it will bring unnecessary worry to the patient. Therefore, the correct detection and diagnosis of iliac vein disease is very important [12].

With the rapid expansion of AI's core technology, the in-depth learning model in the field of medical image diagnosis has been improved. A deep learning mode was established in the recognition of iliac vein compression points based on ultrasound images to realize the classification of the severity of various lesions and automatically identify the disease and effectively help doctors to diagnose and treat it. Due to different compression point sizes, shapes, and textures, the establishment of an accurate and effective recognition model is of specific research value and clinical application value. Since the application of AI in medical treatment, especially the development of deep learning in images, many deep learning methods have been applied to medical image processing. The convolutional neural network (CNN) is the most common network model in image extraction. All effective networks include networks that provide excellent results for daily graphics, including the residual neural network, dense convolutional neural network (DenseNet), Mobile Net, and the top-ranked ImageNet network [13]. However, vein ultrasound images have higher noise and higher volatility compared with ordinary images, and the imaging of the vein end is not obvious. The common network limits the extraction of edges and textures. In addition, the resolution of the traditional convolution kernel gradually decreases as the number of layers increases, which can reduce the acquisition of more detailed position information [14–16]. Hole convolution has a wider field of view under the same convolution kernel size compared with traditional convolution.

A dense multireceptive field convolutional neural network based on AI was proposed in this research. It can detect iliac vein compression lesions efficiently and accurately and can evaluate the effectiveness of contrast-enhanced ultrasound in the diagnosis of iliac vein compression by different methods. In addition, a model that can automatically identify compression points was constructed based on deep learning methods to reduce the workload of clinicians.

## 2. Methods

### 2.1. Research Objects

A total of 280 CVD and DVT inpatients (363 affected limbs) in the hospital from January 2017 to January 2021 were selected as the research objects. There were 194 patients with nonthrombotic CVD (265 limbs), including 126 males and 68 females, aged from 25 to 80 years, with an average age of 40.7 ± 11.24 years. There were 90 patients with DVT (98 limbs), including 45 males and 45 females, aged from 25 to 80 years, with an average age of 60.23 ± 12.15 years. The patient's general information, clinical symptoms, history of intravenous treatment, and thrombus cases were recorded.

Inclusion criteria: (i) clinical inpatients diagnosed with CVD or DVT after vascular surgery and (ii) ultrasound and DSA examination of the iliac vein were performed before surgery or surgical treatment, and no venous related treatment was performed.

Exclusion criteria: (i) other diseases may lead to varicose veins (such as Budd–Chiari syndrome), right heart failure, pelvic tumors, pregnancy, and other lower limb venous insufficiency; (ii) diseases affecting the amount of blood in large amounts of chest, ascites, and hypoproteinemia; and (iii) patients who were allergic to contrast media and cannot be tested with DSA.

Patients were randomly rolled into the AI algorithm imaging group and control group according to ultrasound diagnosis results.

In this study, a total of 284 patients with IVCS met the above inclusion criteria and exclusion criteria. This study had been approved by the medical ethics committee of the hospital, and the families of the patients included in the study had all signed informed consent.

### 2.2. Data Acquisition and Image Analysis

#### 2.2.1. Ultrasonic Data Acquisition

The patient needed to fast for more than eight hours before the ultrasound examination of the iliac vein. The patient was in a supine position with his lower extremities slightly eversion. Two-dimensional ultrasonic imaging (2D-US), color Doppler flow imaging (CDFI), and color Doppler energy imaging (CDE) were performed to analyze the energy imaging, vascular enhancement technology (VET), and pulse wave (PW). The abnormal echo of the iliac vein cavity, stenosis, or dilation was observed, so did the formation of collateral blood circulation, the reflux and abnormal echo of the internal bowel veins, and the expansion of the venous cavity of the lower extremities.

#### 2.2.2. Equipment

A 52000 type Doppler ultrasonic diagnostic device was used. The 4c1 convex array detection frequency was 14 mHz, and the 9l4 linear array detection frequency was 4 × 9 mHz. Philips FD2.0 digital subtraction angiography machine was employed.

### 2.3. Experimental Environment

#### 2.3.1. Convolutional Layer Model Construction

CNN realizes image point extraction through convolutional layers. The convolutional layer requires fewer parameters compared with the fully connected layer (the number of weights does not change with the size of the image). In the convolutional layer, the image convolution operation shares the weight of the network. Therefore, the model does not require separate detectors for the same object, and the network translation is consistent with the input result. The convolution operation is between the first layer and the second layer, and the complete connection operation is between the third layer and the fourth layer.  Figure 1 shows a schematic diagram of a convolutional layer and a fully connected layer. The dense multireceptive field CNN (DMRF-CNN) was utilized to extract features from ultrasound images of thyroid nodules. The method of multiporosity convolution and dense connection was used to extract the features of the nodules and transfer the features. “d-x-conv-y” represents the feature map obtained after this kind of hole convolution, *x* represents the size of the hole rate (*x* ∈ {2,3,4}), and *y* represents the number of convolutional layers. “conv” represents the feature map after the traditional convolution kernel convolution, that is, the convolution kernel with a hole rate of 1, which is equivalent to “d1conv-y.” “Cx” represents different cross-layer connections, and different colors represent the feature maps obtained after convolution kernels with different void ratios. This model realizes the fusion of multiple receptive fields with the help of four convolution kernel fusion methods with different void ratios, which can not only achieve the goal but also reduce the parameters and prevent overfitting to a certain extent. In addition, for each dilated convolution module (Dilated Conv), the convolution module of the 0Darknet network was used. A 3 × 3 convolution kernel was utilized, and then, a batch normalization layer was employed to normalize the feature map to prevent the gradient from disappearing, and finally, the LeakyReLU activation function was used. In the DMRF-CNN, information between various layers is exchanged through dense cross-layer connections. The fusion of deep-level feature maps with shallow-level feature maps can make edge features well recognized.

#### 2.3.2. R-CNN

Figure 2 shows the flowchart of the R-CNN (Region-CNN), which is classified into three stages: generating regions of interest, feature extraction based on convolutional neural networks, and classification and positioning.

Since the R-CNN uses a selective search method to generate about 2,000 regional feature points for each image, accurate data points can be selected and the search space can be reduced in target detection. Therefore, the AlexNet CNN is used to extract the features of the image. Because of the automatic AI of the network, it can learn data processing and gradually improves the accuracy.

#### 2.3.3. Dataset and Evaluation Criteria

The dataset from the hospital physical examination center was utilized to conduct the experiment, and finally, 699 vein images were selected, among which each image contained at least one lesion point. Venous compression images of 34 men and 177 women were extracted. The sample underwent data expansion, and the process included color dithering, changing saturation, exposure, and color. In particular, the aspect ratio of the lesion point may interfere with the judgment of the disease, so the random angle change was not used in this experiment. After zooming in, 10,377 images were obtained.  Figure 3 shows the detailed number of training sets and test sets.

#### 2.3.4. Deep Learning Mode

In this experiment, the compression site of the vein was first obtained, and then, the vein ultrasonic image was edited out with the same size, i.e., 240 × 240. Different models were used to categorize data graphs. In the experiment, the probability gradient descent algorithm was used to upgrade the quality and efficiency. The learning efficiency at the beginning of the experiment was 0.01, the number of iterations was 600, and the final training time of the model was about 4 hours. In addition, the rate of Jitter was set to 0.3 during data amplification. The ultrasonic image was edited and randomly inverted at a rate of 0.3. The chroma and exposure was set to 2.5 and the hue to 0.1 to represent the random generation of the image in the range of 0.05–0.12 tones. A 3070 graphics card (13G memory), 8-core CPU, and 16G memory were used to implement the model and Kersa architecture for training as the experimental environment.

### 2.4. Treatment Methods

#### 2.4.1. Treatment Measures

The patient's physical data and the lower extremity venous ultrasound results were recorded. A lateral thigh artery puncture was performed by the Seldinger method in the supine position, depending on the polymortem level, which was through the affected vein in advance of B ultrasound. The sheath of 6F was inserted. The degree, location, extent, and collateral circulation of iliac vein stenosis were determined by angiography. If the skeleton has severe narrowing in the vein or occlusion of the vein, adjuvant treatment can be done through the spinal canal at the occlusion site. Reconfirming of the angiogram in the inferior great vein was carried out, and severe stenosis or occlusion can be found in images with small openings in the lumen. To open the narrow part of the iliac vein, the loach guide wire was inserted. A V-18 guide wire was used to pass through the occlusion without opening. With the majority of the orbital catheter, the majority of the lesions were detected. After balloon dilation, the lesion segment of angiogram intestinal venous stenosis was less than 50%, the vascular elasticity recovery was reduced to 1/3, or the balloon dilation was performed after peripheral collateral circulation was greatly reduced.

#### 2.4.2. Anticoagulation Therapy and Compression Therapy

To prevent puncture bleeding after intracavitary treatment, sterile gauze and elastic bandage should be used for pressure protection of puncture site and 12 h clinical observation. Anticoagulant therapy referred to a subcutaneous injection of low molecular weight heparin (LMWH) with oral administration of Beritol 10 mg twice daily for three months. For patients with high thrombosis risk factors, this may be extended to six months. Patients needed to wear stretch socks for six months after discharge.

#### 2.4.3. Diagnostic Criteria and Cure Indicators

Ultrasonic diagnostic criteria were as follows. During CT venography of completely obstructed thrombosis, this segment of blood vessel did not develop at all or showed signs of sudden interruption of contrast medium at a certain level. For incomplete obstructed thrombosis, CT venography showed cylindrical or low-density contrast areas with different lengths in the venous lumen, and the edge of the venous lumen may have orbit disease caused by the contrast agent alignment. After mechanization and recanalization, CT venography showed that the venous lumen was irregular, narrow, and multibranched, partly dilated, or even twisted. Collateral circulation was established, and CT venography showed irregular collateral vein development around the obstructed vessel. Physical examination of the affected limb was implemented to assess relief of symptoms associated with venous hypertension in the lower extremity with a venous clinical severity score (VCSS). The VCSS scale includes ten clinical symptoms, such as, pain, varicose veins, venous edema, pigmentation, inflammation, sclerosis, number of ulcers, duration of ulcers, diameter of ulcers, and compression treatment. According to the classification of none, light, medium, and heavy, the corresponding score is 0, 1, 2, and 3. The patency rate of the stent was examined by color Doppler ultrasonography or venography to evaluate the patency of the venous outflow tract.

#### 2.4.4. Follow-Up after Treatment

Hospitalization or telephone appointments were made at 3 months, 6 months, and 1 year. Patients were required to wear stretch socks and take anticoagulants. To assess the VCSS for reducing symptoms associated with venous hypertension of the lower extremities, physical examinations of the limbs were performed. The VCSS included ten clinical symptoms, such as varicose veins, edema of veins, pain, pigmentation, inflammation, sclerosis, number of ulcers, duration of ulcers, and diameter of ulcers. The patency rate of the stent was examined by color Doppler ultrasound or venography, and the smoothness of the venous outflow path was assessed.

### 2.5. Statistical Processing

SPSS 20.0 was employed for statistical analysis. The data were expressed as *n*, and the chi-square test was used for comparison in the same group. The measurement data were expressed as positive and negative standard deviations, and the normality test and the variance homogeneity test were performed before the analysis of the two sets of measurement data. The *t*-test was used for the comparison of the average between the normal groups, and the rank sum test was used to compare the mean between groups for normality. When *p* < 0.005, the difference was statistically significant.

## 3. Results

### 3.1. Evaluation of Hole Convolution

Figure 4 shows the difference comparison of the feature extraction effect of the hole convolution with four different kinds of hole ratios. When the hole ratio was two, the effect was ideal. In addition, the accuracy of vein compression image recognition can be improved to a certain extent by introducing the hole ratio.  Figure 5 shows the segmentation and lesion identification of venous compression ultrasound images.

### 3.2. Comparison between Different Models

Figure 6 shows the segmentation comparison between different models. In the traditional feature extraction method, the recall rate was very high and the accuracy was very low. The deep learning methods improved accuracy compared with traditional feature extraction methods. However, the recall rate and accuracy of these methods had changed a lot, and the stability of model recognition was not good. The recall rate and accuracy of the DMRF-CNN were not significantly different. Therefore, the DMRF-CNN had good stability for identifying venous compression points and achieved good accuracy.  Figure 7 shows the efficiency graph compared with other feature extraction methods.

### 3.3. Technical Success Rate

Sixty-six patients in the two groups successfully completed endovascular treatment for iliac vein stenosis or occlusion. After endovascular treatment, angiography confirmed different degrees of intestinal vein stenosis or occlusion, and the pelvic side blood circulation was significantly reduced. Twenty-three patients with venous flow received a second treatment in the observation group.  Figure 8 shows that there was no statistical difference in the ratio of venous flow between the two groups.

### 3.4. Relief of Intravenous Clinical Symptoms

The analgesic rate of 66 patients in the angiographic group was 88.42% and that in the control group was 86.3%. Most of the symptoms of limb swelling disappeared, and the patients' pain significantly reduced. The swelling rate of the angiographic group was 91.1%, and the swelling rate of the control group was 89.72%. Among patients with compound ulcers, the ulcer cure rate in the observation group was 83.20% in groups with different improvement and cure degrees. The average VCSS score at 3 months after treatment was 11.37 ± 3.12 points, that at 6 months after treatment was 7.98 ± 3.66, that at 12 months after treatment was 7.33 ± 2.12, that at 24 months after treatment was 15.15 ± 4.57, and that at 36 months after treatment was 14.33 ± 2.13. The average VCSS score of each follow-up point was 6.53 ± 2.33, which was lower than that before treatment, and there were statistical differences before and after treatment (*p* < 0.005). Therefore, the treatment method of the angiography group was effective.  Figure 9 shows the comparison of pain relief rates between the two groups.

Comparison of VCSS scores before treatment, 3 months after treatment, and 6 months after treatment between the two groups showed that *p* > 0.005. There was no difference in the severity of intravenous clinical symptoms between the two groups before treatment. The curative effect was equivalent within 6 months. The average score of VCSS at 12 months after treatment, 24 months after treatment, and 36 months after treatment was compared, and there were statistical differences, *p* < 0.005. The average VCSS score of the angiographic group was significantly lower than that of the control group, indicating that the angiographic group had a more significant clinical effect than the control group in the midterm effect at 12, 24, and 36 months.  Figure 10 shows the comparison of VCSS scores between the two groups at 3, 6, 12, 24, and 36 months after treatment.

The VCSS scores before treatment, 3 months after treatment, and 6 months after treatment were compared, and *p* > 0.05. The severity of intravenous clinical symptoms was compared between the two groups within 6 months, and there was no difference between the two groups. The average VCSS score at 12 months after treatment, 24 months after treatment, and 36 months after treatment was compared, and the results showed statistical differences, *p* < 0.005. The average VCSS score of the control group was significantly lower than that of the angiographic group. Significant effects were achieved within 12, 24, and 36 months.  Figure 10 shows the comparison of the VCSS scores of the two groups at 3, 6, 12, 24, and 36 months after treatment.

## 4. Discussion

IVCS is caused by a series of clinical symptoms of pelvic or venous return disorders due to venous pressure and/or an unusual bonding structure. The main manifestations are lower extremity skin pigmentation, lower extremity vein collapse, and spermatic vein flow [17]. MTS was thought to be a rare disease in the past. With the development of imaging techniques and improved understanding of MTS, it has been applied to a variety of lesions; however, the extent of its use is now overrated. Compression of the right common iliac vein is rare and is related to anatomical differences between the bony veins of the two intestines. The high rate of MTS in young women may be related to the obvious lumbar vertebra physiology of women and the long-term use of contraceptives in young women. The extent of enteric venous compression stenosis is not well defined. Collateral circulation may be observed by imaging [18].

With the improvement of people's living standard and the progress of medical technology, many people can get a physical examination at a very low cost. Intravenous compression examination is one of the most common items of physical examination. This has also led to an increase in the detection rate of venous compression syndrome. In addition, the same compression site can be identified with different results, depending on the clinician's clinical judgment. In addition, the gap between urban and rural medical level also makes it difficult for the county hospitals to distinguish compression lesions. Experience is likely to lead to overtreatment of patients [19]. It brings unnecessary pain and burden to patients. To solve this problem, an effective deep learning framework was proposed in this research to help doctors identify and judge the disease.

The general structure flowchart of this method was proposed and compared with other backbone networks based on YOLOV3. The dataset for comparison was from our hospital, and 699 ultrasound images of thyroid nodules were eventually collected. The graph features on the test set and detection time were used to evaluate the validity of the model. Then, YOLOV3-DMRF was verified to have the best detection performance. The graph features reached 91.77% in the dataset collected by myself, and the detection time was 4.2 seconds. In the open dataset, the mapping reached 94.72%, and the detection time was 2.3 seconds. To prove the feature extraction effect of the DMRF-CNN, the classification performance of the DMRF-CNN was compared with that of other AI networks. Finally, it was proved that the DMRF-CNN was superior to other CNNs in classification performance based on different evaluation criteria.

## 5. Conclusion

The contrast-enhanced ultrasound images were used in the treatment of venous compression syndrome. Compared with the lesion site manually delineated by the doctor on the angiography image, the method proposed in this study had little difference in both the therapeutic effect and the convenience of operation. This method significantly shortened the time needed for outlining compared with traditional manual segmentation. In the future, it needs to verify the performance of our model in more centers, CEUS models, and more disease types. In addition, to study various parameters of image formation based on this method, its clinical diagnosis and prognosis prediction need to be further studied.

## Figures and Tables

**Figure 1:** Schematic diagram of the convolutional layer and fully connected layer.

**Figure 2:** Flowcharts of the R-CNN.

**Figure 3:** Detailed number of the training set and test set.

**Figure 4:** The influence of four kinds of hole convolutions on the feature extraction effect (1, 2, 3, and 4 represent four kinds of hole rate labels).

**Figure 5:** The effect of hole convolution on feature extraction (The red parts are the focus points extracted by the artificial intelligence algorithm, and the three images are from three randomly selected patients).

**Figure 6:** Traditional extraction method (a) and DMRF-CNN extraction (b) (the red parts are the focus points extracted by the artificial intelligence algorithm).

**Figure 7:** Accuracy and precision comparison with other model extraction methods.

**Figure 8:** The proportion of varicose veins in the two groups.

**Figure 9:** Comparison of pain relief rates between the two groups.

**Figure 10:** Comparison of VCSS scores between the two groups at 3, 6, 12, 24, and 3 months after treatment. ^*∗*^Significance of the difference.

## Data Availability

The data used to support the findings of this study are available from the corresponding author upon request.
